The article "Mechanisms of nanosized titanium dioxide-induced testicular oxidative stress and apoptosis in male mice" was retracted in 2015. Reasons: errors in the analysis; errors in the methods; duplicated images.

# Mechanisms of nanosized titanium dioxide-induced testicular oxidative stress and apoptosis in male mice

**DOI:** 10.1186/s12989-014-0047-3

**Published:** 2014-09-12

**Authors:** Xiaoyang Zhao, Lei Sheng, Ling Wang, Jie Hong, Xiaohong Yu, Xuezi Sang, Qingqing Sun, Yuguan Ze, Fashui Hong

**Affiliations:** 1 Medical College of Soochow University, Suzhou 215123, China; 2 Library of Soochow University, Suzhou 215123, China; 3 Jiangsu Province Key Laboratory of Stem Cell Research, Soochow University, Suzhou 215007, China; 4 Cultivation base of State Key Laboratory of Stem Cell and Biomaterials built together by Ministry of Science and Technology and Jiangsu Province, Suzhou 215007, China

**Keywords:** Titanium dioxide nanoparticles, Testis, Oxidative stress, Sertoli cell apoptosis, Gene expression

## Abstract

**Background:**

Due to the increased application of titanium dioxide nanoparticles (TiO_2_ NPs) in the food industry and daily life, their potential toxic effects in humans and animals have been investigated. However, very few studies have focused on testicular oxidative stress and/or apoptosis.

**Methods:**

In order to understand the possible molecular mechanisms of testicular lesions following exposure to TiO_2_ NPs, male mice were exposed to 2.5, 5, or 10 mg/kg body weight TiO_2_ NPs for 90 consecutive days. Testicular oxidative stress and apoptosis were then evaluated, and the testicular mRNA expression of several genes and their proteins involved in oxidative stress and/or apoptosis was investigated.

**Results:**

TiO_2_ NPs entered Sertoli cells and caused severe testicular oxidative damage and/or apoptosis, accompanied by excessive production of reactive oxygen species and peroxidation of lipids, proteins and DNA as well as a significant reduction in antioxidant capacity. Furthermore, exposure to TiO_2_ NPs resulted in the up-regulation of caspase-3, Nrbp2, and cytochrome c expression, and caused down-regulation of SOD, CAT, GPx, GST, GR, Cyp1b1, Car3, Bcl-2, Acaa2, and Axud1 expression in mouse testis.

**Conclusions:**

TiO_2_ NPs entered Sertoli cells via the blood-testis barrier and were deposited in mouse seminiferous cord and/or Sertoli cells, causing oxidative damage and apoptosis.

## 1 Background

The use of nanosized materials in consumer and industrial products has increased due to their distinctive physicochemical properties, including high reactivity, color changes, lower melting temperature, and greater solar radiation absorption. In particular, titanium dioxide nanoparticles (TiO_2_ NPs) have been used in crop production, dietary supplements, food additives, food packaging components, medicine, toothpastes, sunscreens, cosmetics, and waste water treatment [1]-[11]. This widespread use of TiO_2_ NPs has inevitably led to harmful biological responses in humans, and animals [12], particularly in the reproductive system [13].

The article "Mechanisms of nanosized titanium dioxide-induced testicular oxidative stress and apoptosis in male mice" was retracted in 2015. Reasons: errors in the analysis; errors in the methods; duplicated images.

Komatsu et al. suggested that TiO_2_ NPs could migrate to Leydig cells, decrease the viability and proliferation of these cells, and increase the gene expression levels of heme oxygenase-1 and steroidogenic acute regulatory protein of Leydig cells in mouse testis *in vitro*[14]. Hou et al. reported that exposure to TiO_2_ NPs led to obvious morphological changes in follicles, a reduction in follicle survival, reduced formation of antral follicles, and inhibition of rat follicle development and oocyte maturation *in vitro*[15]. Suzuki et al. found that TiO_2_ NPs entered the cytoplasm of cultured Chinese hamster ovary cells, but not the nucleus [16]. Di Virgilio et al. observed significant agglomeration of TiO_2_ NPs on both the plasma membrane and the cytoplasm inducing genotoxic and cytotoxic effects [17]. Exposure to TiO_2_ NPs can occur via inhalation, transdermal absorption, and ingestion, therefore, the ovaries and testes may also be target organs of toxicity in mammals exposed to TiO_2_ NPs. The importance of TiO_2_ NP exposure has been highlighted in *in vivo* studies. Ema et al. indicated that TiO_2_ NPs injected subcutaneously into pregnant mice resulted in male offspring with altered spermatogenesis and histopathological changes in the testes [18]. Takeda et al. also studied pregnant mice injected subcutaneously with TiO_2_ NPs, and TiO_2_ NPs were observed to migrate to spermatids, Sertoli cells and Leydig cells in the male offspring, resulting in disorganization in seminiferous tubules and reductions in daily sperm production, sperm motility and Sertoli cell number [19]. Male mice exposed to TiO_2_ NPs by intraperitoneal injection showed marked reductions in sperm numbers and motility, and elevated abnormal sperm and germ cell apoptosis in the testis [20]. Our recent studies demonstrated that TiO_2_ NPs can migrate to the ovary and testis, resulting in injury, a reduction in fertility, lower sperm concentration and sperm motility, higher malformation rates of sperm, and alterations in the gene expression profile in the damaged ovaries and testes in mice [21],[22]. Many conditions or events associated with male infertility can induce oxidative stress and germ cell apoptosis. Given that spermatozoa are rich in polyunsaturated fatty acids, they are very susceptible to attack by reactive oxygen species (ROS) [23],[24], while protection from lipid peroxidation is mainly due to the activity of glutathione peroxidase (GPx), an enzyme important for maintaining sperm motility and viability [25],[26]. The reproductive system of male mammals mainly consists of the testis, epididymis and ductus deferens. The testis produces spermatozoa and the epididymis stores the spermatozoa and completes sperm maturation. We hypothesize that decreased sperm motility and viability caused by exposure to TiO_2_ NPs may be associated with testicular oxidative stress and/or apoptosis. To date, no studies have examined whether TiO_2_ NPs induce testicular oxidative stress and/or apoptosis by assessing the antioxidant capacity, and alterations in oxidative stress and/or apoptosis-related gene expression in male mice. Thus, the aims of the present study were to test the hypothesis that TiO_2_ NPs induce oxidative stress and/or apoptosis in the testis of mice by causing a reduction in antioxidant capacity and alterations in oxidative stress and/or apoptosis-related gene expression. In addition, the mechanisms of TiO_2_ NP-induced oxidative stress and/or apoptosis in mouse testis were evaluated.

The article "Mechanisms of nanosized titanium dioxide-induced testicular oxidative stress and apoptosis in male mice" was retracted in 2015. Reasons: errors in the analysis; errors in the methods; duplicated images.

## 2 Results

### 2.1 TiO_2_ NPs characteristics

XRD measurements showed that TiO_2_ NPs exhibited the anatase structure (Figure 1), and the average particle size calculated from the broadening of the (101) XRD peak of anatase was approximately 5.5 nm using Scherrer’s equation. TEM demonstrated that the average size of the powder particles (Figure 2a) and NPs suspended in HPMC solvent after incubation ranged from 5—6 nm, respectively (Figure 2b), which was consistent with the XRD results. The sample surface area was generally smaller than that estimated from the particle size, and it would seem that aggregation of the particles may have caused this decrease. To confirm the dispersion and stability of the TiO_2_ NP suspension, the aggregated size and the ζ potential of TiO_2_ NPs in HPMC were measured. Following 12, 18, and 24 h incubation, the mean hydrodynamic diameter of TiO_2_ NPs in HPMC solvent ranged from 210 to 450 nm (mainly 310 nm), as measured by DLS, which indicated that the majority of TiO_2_ NPs were clustered and aggregated in solution. In addition, the ζ potential was 7.57, 8.53, and 9.28 mV, respectively.

**Figure 1:** **The (101) X-ray diffraction peak of anatase TiO**_**2**_**NPs.** The average particle size was about 5 nm calculated using Scherrer’s equation.

**Figure 2:** **Transmission electron microscope images of anatase TiO**_**2**_**NPs. (a)** TiO_2_ NP powder; **(b)** TiO_2_ NPs suspended in HPMC solvent after incubation for 12 h. TEM images showed that the sizes of the TiO_2_ NP powder or TiO_2_ NPs suspended in HPMC solvent for 12 h ranged from 5 to 6 nm, respectively.

### 2.2 Histopathological evaluation

The histological changes in the testis specimens are shown in Figure 3. Unexposed testicular samples showed normal histology. The seminiferous tubules in these samples showed numerous spermatogonia, primary spermatocytes, secondary spermatocytes, spermatids, spermatozoids, Sertoli cells and Leydig cells (Figure 3). However, the samples from the mice exposed to TiO_2_ NPs exhibited the following severe pathological changes: a significant reduction in the thickness of the germinal layer, a reduction in the number of spermatogonia, rupture of the seminiferous tubules, vacuolation, spermatocyte and Sertoli cell apoptosis or necrosis, and irregular arrangement of spermatocytes and Sertoli cells in the seminiferous tubules (Figure 3). In addition, we also observed a significant number of black agglomerates in the seminiferous tubules exposed to 10 mg/kg of TiO_2_ NPs (Figure 3). Confocal Raman microscopy further showed a characteristic TiO_2_ peak in the black agglomerates (148 cm^−1^), which further confirmed the deposition of TiO_2_ in the testis (see Raman intensity insets in Figure 3).

The article "Mechanisms of nanosized titanium dioxide-induced testicular oxidative stress and apoptosis in male mice" was retracted in 2015. Reasons: errors in the analysis; errors in the methods; duplicated images.

**Figure 3:** **Histopathological observations of mouse testis following intragastric administration of TiO**_**2**_**NPs for 90 consecutive days.** The blue circle indicates few sperm, breakages or vacuolation, the yellow circle indicates apoptosis and/or necrosis of Sertoli cells, and the blue arrow indicates damaged seminiferous tubule. The red arrows indicate vacuolation, the yellow arrows indicate irregular arrangement of Sertoli cells, and the red circle indicates black agglomerates in the testis. The green arrow spot denotes a representative cell loaded with TiO_2_ NPs. The right panel shows the corresponding Raman spectra identifying specific peaks at about 148 cm^−1^.

### 2.3 Sperm morphology

As shown in Figure 4, exposure to TiO_2_ NPs induced abnormalies in the sperm head and tail. Head abnormalities included amorphous, hookless, banana-shaped and double-headed sperm. TiO_2_ NPs also caused the formation of folded, coiled, bent and double-tailed sperm. In addition to these morphological alterations, many sperm tails appeared in the smears of treated mice with detached heads. Sperm also showed an acute bend at the cephalocaudal junction from which fibrils projected out.

**Figure 4:** **Morphological changes in mouse sperm following intragastric administration of TiO**_**2**_**NPs for 90 consecutive days.**

### 2.4 Sertoli cell ultrastructure

Changes in the cell ultrastructure in mouse testicular samples are shown in Figure 5. Sertoli cells in the control group contained elliptical nuclei with homogeneous chromatin (Figure 5); however, cell ultrastructure in mouse testicular tissue treated with TiO_2_ NPs indicated typical apoptosis, including significant mitochondrial swelling and cristae disappearance, nuclear membrane collapse and chromatin marginalization (Figure 5). In addition, we also observed a significant number of black agglomerates in the cytoplasm and/or nucleus in the TiO_2_ NP-exposed testicular tissues (Figure 5). Confocal Raman microscopy showed a characteristic TiO_2_ NP peak in the black agglomerate (148 cm^−1^), which further demonstrated the aggregation of TiO_2_ NPs in cells (see the Raman intensity insets in Figure 5). These results suggested that chronic exposure to TiO_2_ NPs resulted in Sertoli apoptosis in the testis, which may be due to excessive ROS production and increased peroxidation levels.

The article "Mechanisms of nanosized titanium dioxide-induced testicular oxidative stress and apoptosis in male mice" was retracted in 2015. Reasons: errors in the analysis; errors in the methods; duplicated images.

**Figure 5:** **Ultrastructure of Sertoli cells in mouse testis caused by intragastric administration of TiO**_**2**_**NPs for 90 consecutive days.** The yellow arrow indicates mitochondrial swelling, blushing, and/or cristae disappearance, the green arrow indicates TiO_2_ NP aggregation in mitochondria, and the red arrow indicates nuclear membrane collapse and chromatin marginalization in Sertoli cells. The green arrow spot denotes a representative cell loaded with TiO_2_ NPs. The right panel shows the corresponding Raman spectra identifying specific peaks at about 148 cm^−1^.

### 2.5 Oxidative damage of testis

To confirm the molecular mechanism of TiO_2_ NP-induced oxidative stress and/or apoptosis of testicular cells, oxidative indices including O_2_^**·−**^, H_2_O_2_, MDA, PC as well as 8-OHdG levels were examined. As shown in Table 1, O_2_^**·−**^, H_2_O_2_, MDA, and PC levels were significantly elevated and increased with increasing TiO_2_ NPs dose (P < 0.05). A marked increase in testicular 8-OHdG level was observed in the TiO_2_ NP-treated groups (P < 0.05 or 0.01), indicating that excessive ROS production led to DNA damage in the testis due to TiO_2_ NP–induced toxicity.

**Table 1:** **Oxidative stress in testis of male mice caused by intragastric administration with TiO**_**2**_**NPs for 90 consecutive days**

**Oxidative stress**	**TiO**_**2**_**NPs (mg/kg BW)**			
	**0**	**2.5**	**5**	**10**
O_2_^.-^ (nmol/mg prot⋅min)	45 ± 2.42	57 ± 2.96*	78 ± 4.28**	103 ± 5.29***
H_2_O_2_ (nmol/mg prot⋅min)	63 ± 3.49	73 ± 3.82*	95 ± 4.86**	125 ± 6.36***
MDA (nmol/ mg prot)	570 ± 29.62	1030 ± 51.72*	1880 ± 95.08**	2580 ± 130.55***
PC (nmol/mg prot)	960 ± 48.75	1170 ± 58.93*	2220 ± 112.56**	4070 ± 205.57***
8-OHdG (ng/g tissue)	310 ± 15.86	3390 ± 169.78*	6380 ± 320.81**	8660 ± 435.63***

*p < 0.05, **p < 0.01, and ***p < 0.001. Values represent mean ± SD (*N* = 5).

### 2.6 Antioxidant defense

The activities of antioxidative enzymes in the testis, including SOD, CAT, APx, GR and GST were examined (Table 2). These enzymes in testes exposed to TiO_2_ NPs were significantly decreased with increasing TiO_2_ NP dose (Table 2, P < 0.05). To further explore the effects of TiO_2_ NP stress on antioxidant capacity, the contents of GSH and ascorbic acid in the testis were examined and are shown in Table 2. Marked decreases in GSH and ascorbic acid in the three TiO_2_ NP-treated groups were observed (P < 0.05). These results suggested that exposure to TiO_2_ NPs resulted in decreased ROS removal in mouse testis.

The article "Mechanisms of nanosized titanium dioxide-induced testicular oxidative stress and apoptosis in male mice" was retracted in 2015. Reasons: errors in the analysis; errors in the methods; duplicated images.

**Table 2:** **Alterations of antioxidative capacity in mouse testis after intragastric administration with TiO**_**2**_**NPs for 90 consecutive days**

**Enzyme activity**	**TiO**_**2**_**NPs (mg/kg BW)**			
	**0**	**2.5**	**5**	**10**
SOD (unit/mg protein⋅min)	51 ± 2.71	35 ± 1.79*	23 ± 1.39**	13 ± 0.72***
CAT (unit/mg protein⋅min)	73 ± 3.82	53 ± 2.79*	35 ± 1.86**	25 ± 1.39***
GSH-Px (unit/mg protein⋅min)	57 ± 2.96	43 ± 2.29*	29 ± 1.56**	18 ± 1.15***
GST (unit/mg protein⋅min)	50 ± 2.65	37 ± 2.06*	22 ± 1.2**	15 ± 0.8***
GR (unit/mg protein⋅min)	59 ± 3.23	50 ± 2.65*	36 ± 1.85**	29 ± 1.56***
GSH (ng/g tissue)	2360 ± 118.56	1910 ± 95.53*	1090 ± 55.56**	510 ± 25.68***
Ascorbic acid (ng/g tissue)	2050 ± 103.28	1480 ± 75.22*	850 ± 43.55**	420 ± 22.67***

*p < 0.05, **p < 0.01, and ***p < 0.001. Values represent mean ± SD (*n* = 5).

### 2.7 Assay of gene and protein expression

In the present study, GDPH was chosen as the endogenous control gene. The expression level of the GDPH gene was constant, with an expression ratio of almost one in all the samples (data not listed). Therefore, using this gene as a reference, changes in the expression levels of the 13 oxidative stress and/or apoptosis-related genes were evaluated and compared following exposure to TiO_2_ NPs for 90 consecutive days (Figure 6). The expression levels of SOD, CAT, GPx, GST, GR, Cyp1b1, Car3, Bcl-2, Acaa2, and Axud1 decreased gradually, whereas the expression levels of caspase-3, Nrbp2, and cytochrome c increased significantly in mouse testis with increasing TiO_2_ NP dose (P < 0.05 or 0.01), respectively. TiO_2_ NP-induced oxidative stress and/or apoptosis-related molecule expression was also examined at the protein level following exposure to various doses of TiO_2_ NPs for 90 consecutive days (Figure 7). ELISA showed that TiO_2_ NPs caused significant reductions in SOD, CAT, GPx, GST, GR, Cyp1b1, Car3, Bcl-2, Acaa2, and Axud1 protein expression, and elevated the levels of caspase-3, Nrbp2, and cytochrome c protein expression in mouse testis (P < 0.05 or 0.01), respectively.

The article "Mechanisms of nanosized titanium dioxide-induced testicular oxidative stress and apoptosis in male mice" was retracted in 2015. Reasons: errors in the analysis; errors in the methods; duplicated images.

**Figure 6:** **Alterations in the mRNA expression of oxidative stress and/or apoptosis-related genes in mouse testis caused by intragastric administration of TiO**_**2**_**NPs for 90 consecutive days.** *p < 0.05, **p < 0.01, and ***p < 0.001. Values represent mean ± SD (*n* = 5).

**Figure 7:** **Alterations in the expression of oxidative stress and/or apoptosis-related proteins in mouse testis caused by intragastric administration of TiO**_**2**_**NPs for 90 consecutive days.** *p < 0.05, **p < 0.01, and ***p < 0.001. Values represent mean ± SD (*n* = 5).

These results are consistent with the histological findings and Sertoli cell ultrastructure in the testicular sections observed in the treated mice.

## 3 Discussion

Studies on the oxidative impairments in the male reproductive system in animals due to nanosized materials are limited. In addition, it is not known whether TiO_2_ NPs enter Sertoli cells inducing oxidative disturbances and/or apoptosis, and the mechanisms involved have not been defined. This has relevance as elevated oxidative stress in the testicular milieu was demonstrated to have profound implications for testicular physiology and sperm function following exposure to nanosized materials [13],[24],[27].

Oxidative damage can affect many classes of molecules including lipids, proteins, nucleic acids, and sugars. Thus, the cell nucleus, mitochondrial membranes, structural and cytoplasmic proteins, complex carbohydrates, RNA, and DNA may all potentially be affected by oxidative stress [28]. In testicular tissue with high rates of metabolism and cell replication, oxidative stress can be especially damaging, making the antioxidant capacity of the tissue very important. Our data revealed that TiO_2_ NPs crossed the blood–testis barrier and were deposited in the seminiferous cord, were translocated to Sertoli cells and/or the nucleus, and caused severe pathological changes such as few sperm, sperm breakage, rupture of the seminiferous tubules, vacuolation, irregular arrangement of Sertoli cells, apoptosis, and significant oxidative impairment in the mouse testis. The pathological changes in the testis were similar to those in our previous report [22]. However, Guo et al. suggested that male mice exposed to rutile TiO_2_ NPs (30 nm) or ZnO NPs (30 nm) by intraperitoneal injection for one week showed significantly increased germ cell apoptosis in the testis without exhibiting significant testicular and/or epididymal lesions [20],[29]. Bai et al. suggested that repeated intravenous injections of water-soluble multi-walled carbon nanotubes (20–30 nm) in male mice for 15 days caused oxidative stress in the testis without affecting fertility, and the oxidative stress and testicular damage were repaired by day 60 and 90, respectively [27]. Exposure to black carbon NPs was demonstrated to increase partial vacuolation of the seminiferous tubules [30]. Furthermore, mice intravenously injected with amorphous nanosilica particles (70 nm) for one week, confirmed that the NPs penetrated the blood–testis barrier and the nuclear membranes of spermatocytes, but did not produce any apparent testicular injuries in male mice [31]. We consider that the inconsistent findings from these reports may be due to the different NPs type, size, exposure time, and particularly clearance rates from the circulation and tissues.

The article "Mechanisms of nanosized titanium dioxide-induced testicular oxidative stress and apoptosis in male mice" was retracted in 2015. Reasons: errors in the analysis; errors in the methods; duplicated images.

Evidence in favor of our central hypothesis was the enhanced levels of MDA, PC and 8-OHdG, as well as ROS levels, and decreased antioxidative enzyme activities including SOD, CAT, GPx, GR and GST and antioxidant contents such as GSH and ascorbic acid in the testes due to TiO_2_ NP exposure. The occurrence of oxidative impairments in the testis raises the question as to whether this effect could be interpreted as a primary effect of TiO_2_ NPs in the testis as TiO_2_ NPs are known prooxidants and their potential to generate free radicals, damage DNA, and induce apoptosis/necrosis is well documented *in vitro*[32] and *in vivo*[33]. While, it is difficult to precisely answer this question based on the data obtained in the current study, it can be reasonably postulated that TiO_2_ NPs do cause significant oxidative stress in mouse testis.

TiO_2_ NP-induced oxidative damage in the testis responded to modulation of antioxidant capacity. Decreased antioxidant enzymes, ascorbic acid and GSH markedly aggravated TiO_2_ NPs induced oxidative damage in the testis as shown by elevated MDA and ROS levels in the cytosol and mitochondria. The major antioxidant enzymes in mammals are SOD, CAT, and GPX, the latter necessitating a number of other enzymes, e.g. GR and GST, required for the recycling or elimination of GSH. All of these antioxidant enzymes are expressed in the testis [34]-[36]. SOD converts O_2_^**·−**^ to H_2_O_2_ and O_2_, and CAT and GPX reduce H_2_O_2_ to H_2_O and O_2_. GR reduces glutathione disulfide (GSSG) to the sulfhydryl form, GSH, which is an important cellular antioxidant. Elevated GR activity can increase the GSH/GSSG ratio, which is required for ascorbic acid regeneration [37]. Furthermore, GST, previously known as ligandin, is from a family of eukaryotic and prokaryotic phase II metabolic isozymes best known for their ability to catalyze the conjugation of GSH to xenobiotic substrates for the purpose of detoxification [38]. In the present study, our data suggest that exposure to TiO_2_ NPs significantly decreased the activities of SOD, CAT, GPX, GR, and GST, and their gene and protein levels, resulting in a higher level of ROS production, increased ROS toxicity, testicular tissue and cell damage in male mice following exposure to TiO_2_ NPs. A number of non-enzyme factors also function as antioxidants in the testis. Of these, ascorbic acid and GSH have proven efficacy in reducing testicular oxidative stress by removing ROS either directly or indirectly by being involved in the ascorbic acid–GSH cycle under different conditions [39]-[43]. Ascorbic acid is considered to be a major antioxidant in the testis, and neutralizes ROS and prevents sperm agglutination. It is an electron donor in redox systems, prevents lipid peroxidation, recycles vitamin E and protects against DNA damage induced by the hydrogen peroxide radical [44]. Oral administration of 200 mg of ascorbic acid together with vitamin E and GSH for a period of 2 months significantly reduced hydroxyguanine (8-OH-dG) levels in spermatozoa and increased the sperm count [45]. In the present study, however, the depletion of ascorbic acid and GSH in the testis caused by TiO_2_ NPs was associated with increases in ROS, MDA, PC, and 8-OH-dG, suggesting that the testis was using antioxidant defenses to prevent oxidative stress, which caused severe oxidative damage in the mouse testis. The oxidative damage and reductions in antioxidants caused by TiO_2_ NPs were consistent with those in mouse liver [46], kidney [47],[48], lung [49],[50], brain [51], and ovary [21].

The article "Mechanisms of nanosized titanium dioxide-induced testicular oxidative stress and apoptosis in male mice" was retracted in 2015. Reasons: errors in the analysis; errors in the methods; duplicated images.

The blood-testis barrier is formed by the tight junctions of Sertoli cells [52]. Therefore, TiO_2_ NP deposition in the testis is closely related to seminiferous tubule injury or apoptosis of Sertoli cells following exposure to TiO_2_ NPs. To understand the mechanisms of oxidative stress and/or apoptosis, the expression of oxidative stress and/or apoptosis-related genes and their proteins in the testis was detected and is listed in Figures 6 and 7. Of the genes involved in apoptosis and/or oxidative stress, caspase-3, Nrbp2, and cytochrome c were markedly up-regulated, while Cyp1b1, Car3, Bcl-2, Acaa2, Axud1, SOD, CAT, GPX, GR, and GST were significantly down-regulated in the mouse testis. Caspase-3 is activated in the apoptotic cell both by extrinsic (death ligand) and intrinsic (mitochondrial) pathways [53]-[56]. It has been reported that TiO_2_ NPs induced apoptosis in mouse spleen by activating caspase-3 [57]. The present study showed that caspase-3 expression in mouse testis was increased, in concordance with the above-mentioned report on the effects of TiO_2_ NPs in mouse spleen. Overexpression of Bcl-2 prevents cells from undergoing apoptosis in response to a variety of stimuli. Cytosolic cytochrome c is necessary for initiation of the apoptotic program, suggesting a possible connection between Bcl-2 and cytochrome c, which is normally located in the mitochondrial intermembrane space. Cells undergoing apoptosis were found to have elevated cytochrome c in the cytosol and a corresponding decrease in the mitochondria. Overexpression of Bcl-2 prevented the efflux of cytochrome c from the mitochondria and the initiation of apoptosis [58],[59]. In the present study, Bcl-2 expression was significantly decreased, whereas cytochrome c was markedly increased in the TiO_2_ NP-exposed mouse testis, suggesting that Bcl-2 may play an important role in TiO_2_ NP-induced Sertoli apoptosis in the mouse testis. These results were similar to those of TiO_2_ NPs-induced apoptosis in mouse spleen [60]. Nrbp2 belongs to the protein kinase superfamily, and was found to be expressed in a subset of tumor cells in human medulloblastoma and protected nestin-positive neural progenitors against apoptosis during differentiation [61]. Nrbp2 upregulation in the mouse testis may prevent Sertoli cell apoptosis and may be a response to TiO_2_ NP-induced toxicity. Cao et al. indicated that Acaa2 abolished Bc1-2/adenovirus E1B 19 kD-interacting protein 3 (BNIP3)-mediated apoptosis and mitochondrial damage [62]. *Axud1* is a member of the gene family encoding nuclear proteins which contain cysteine- and serine-rich domains, and is often considered to be related to reduced apoptosis [63]. Therefore, Sertoli apoptosis in testicular tissue caused by TiO_2_ NPs may be due to a marked reduction in Acaa2 and Axud1 expression. Of the genes and their proteins involved in oxidative stress, SOD, CAT, APX, GR, and GST were highly suppressed. SOD catalyses the dismutation of superoxide anion by successive oxidation-reduction of the transition metal at the enzyme’s active site [64]. CAT converts hydrogen peroxide to hydrogen and water. GPX catalyzes the breakdown of H_2_O_2_ and organic hydroperoxides. GPX can directly reduce phospholipid hydroperoxides inside biological membranes to lipid and water, and is essential for survival and important in repairing damage due to lipid peroxidation [65]. GPX also protects against mitochondrial apoptosis and decreases in mitochondrial ATP generation in the presence of oxidative stress, and is strongly expressed in the mitochondria of testis and spermatozoa [66],[67]. GR plays a key role in oxidative stress by converting GSSG to GSH. Increased GR activity can elevate the GSH/GSSG ratio, which is required for ascorbic acid regeneration [37]. GST is able to conjugate GSH to the toxic reactive compounds, 4-hydroxynonenal and cholesterol α-oxide, which are generated during the oxidation of membranes. The GPx activity of some GST proteins also suggests that they may be important in the detoxification of organic hydroperoxides [68]. Thus, decreased expression of SOD, CAT, GPX, GR, and GST in the mouse testis aggravated TiO_2_ NP–induced oxidative stress. Car3 has been demonstrated to rapidly glutathionylate *in vivo* and *in vitro* when cells are exposed to oxidative stress, and it is one of the most carbonylated proteins in rodent liver [69]. Overexpression of Car3 decreased steady-state levels of intracellular ROS, increased the proliferation rate, and protected cells against H_2_O_2_-induced apoptosis [69]. Cyp1b1 is a member of the cytochrome P450 family of proteins and can remove cellular oxygenation products which induce oxidative stress, while a lack of Cyp1b1 increases oxidative stress *in vivo* and *in vitro*[70]. Therefore, the generation of oxidative stress in the TiO_2_ NP–exposed mouse testis may also be closely associated with significant reductions in Car3 and Cyp1b1 expression and removal of ROS.

The article "Mechanisms of nanosized titanium dioxide-induced testicular oxidative stress and apoptosis in male mice" was retracted in 2015. Reasons: errors in the analysis; errors in the methods; duplicated images.

In summary, TiO_2_ NPs entered Sertoli cells via the blood-testis barrier and were deposited in mouse testicular tissue and/or Sertoli cells, causing testicular oxidative damage and cell apoptosis. Furthermore, testicular damage following exposure to TiO_2_ NPs may be related to significant overproduction of ROS, peroxidation of lipids, proteins and DNA, and a significant reduction in antioxidant capacity. Sertoli cell apoptosis caused by TiO_2_ NPs was associated with up-regulation of caspase-3, Nrbp2, and cytochrome c expression, and down-regulation of SOD, CAT, GPx, GST, GR, Cyp1b1, Car3, bcl-2, Acaa2, and Axud1 expression in mouse testis. Therefore, the application of TiO_2_ NPs should be performed with caution to reduce potential risks to humans.

## 4 Materials and methods

### 4.1 Chemicals

Anatase TiO_2_ nanoparticles were prepared via controlled hydrolysis of titanium tetrabutoxide. The details of TiO_2_ NP synthesis were previously described [71],[72]. Hydroxypropylmethylcellulose (HPMC) 0.5% w/v was used as a suspending agent. TiO_2_ powder was dispersed onto the surface of a 0.5% w/v HPMC solution, and then the suspension containing TiO_2_ particles was treated ultrasonically for 15–20 min and mechanically vibrated for 2 or 3 min.

The particle sizes of both the powder and nanoparticles suspended in 0.5% w/v HPMC solution (5 mg/L) following incubation were determined using a TecnaiG220 transmission electron microscope (TEM) (FEI Co., USA) operating at 100 kV, respectively. In brief, particles were deposited in suspension onto carbon film TEM grids, and allowed to air-dry. The mean particle size was determined by measuring > 100 randomly sampled individual particles. X-ray-diffraction (XRD) patterns of TiO_2_ NPs were obtained at room temperature with a charge-coupled device (CCD) diffractometer (Mercury 3 Versatile CCD Detector; Rigaku Corporation, Tokyo, Japan) using Ni-filtered Cu Kα radiation. The average aggregate or agglomerate size of the TiO_2_ NPs after incubation in 0.5% w/v HPMC solution (5 mg/L) for 0, 12 and 24 h was measured by dynamic light scattering (DLS) using a Zeta PALS + BI-90 Plus (Brookhaven Instruments Corp., USA) at a wavelength of 659 nm. The scattering angle was fixed at 90°.

The article "Mechanisms of nanosized titanium dioxide-induced testicular oxidative stress and apoptosis in male mice" was retracted in 2015. Reasons: errors in the analysis; errors in the methods; duplicated images.

### 4.2 Ethics statement

All experiments were conducted during the light phase, and were approved by the Animal Experimental Committee of Soochow University (Grant 2111270) in accordance with the National Institutes of Health Guidelines for the Care and Use of Laboratory Animals (NIH Guidelines).

### 4.3 Animals and treatment

One hundred sixty CD-1 (ICR) male mice (24 ± 2 g) were purchased from the Animal Center of Soochow University (China). The mice were housed in stainless steel cages in a ventilated animal room. The room temperature in the housing facility was maintained at 24 ± 2°C, with a relative humidity of 60 ± 10% and a 12-h light/dark cycle. Distilled water and sterilized food were available *ad libitum*. Before treatment, the mice were acclimated to this environment for five days. All the animals were handled in accordance with the guidelines and protocols approved by the Care and Use of Animals Committee of Soochow University (China).

TiO_2_ NP powder was dispersed onto the surface of 0.5% w/v HPMC and the suspension containing TiO_2_ NPs was treated ultrasonically for 30 min and mechanically vibrated for 5 min. The mice were randomly divided into four groups (*n* = 40 in each group), including a control group treated with 0.5% w/v HPMC and three experimental groups treated with 2.5, 5, or 10 mg/kg TiO_2_ NPs. The mice were weighed, a volume of TiO_2_ NP suspension was calculated for each mouse, and the fresh TiO_2_ NP suspension was administered by gavage using a gavage needle each day for 90 days. Symptoms, growth status, eating, drinking, activity and mortality were observed and carefully recorded daily during the 90-day period. After 90 days, the mice were weighed, anesthetized using ether, and then sacrificed. The testes were quickly removed, placed on ice, dissected, and then frozen at −80°C (except those for histopathological examination).

### 4.4 Histopathological examination of testis

All histopathological tests were performed using standard laboratory procedures [73]. Five sets of testicular tissues from 5 mice were embedded in paraffin blocks, sliced into 5 μm thick sections and then placed onto glass slides (five slices from each testis). Following hematoxylin–eosin staining, the slides were observed and photographed using an optical microscope (Nikon U-III Multi-point Sensor System, USA). The pathologist was blind to the identity and analysis of the pathology slides.

The article "Mechanisms of nanosized titanium dioxide-induced testicular oxidative stress and apoptosis in male mice" was retracted in 2015. Reasons: errors in the analysis; errors in the methods; duplicated images.

### 4.5 Observation of testis ultrastructure

Testes (*n* = 5 in each group) were fixed in a fresh solution of 0.1 M sodium cacodylate buffer containing 2.5% glutaraldehyde and 2% formaldehyde followed by a 2 h fixation period at 4°C with 1% osmium tetroxide in 50 mM sodium cacodylate (pH 7.2-7.4). Staining was performed overnight with 0.5% aqueous uranyl acetate. The specimens were dehydrated in a graded series of ethanol (75, 85, 95, and 100%), and embedded in Epon 812. Ultrathin sections were obtained, contrasted with uranyl acetate and lead citrate, and observed with a HITACHI H600 TEM (HITACHI Co., Japan). Testicular apoptosis was determined based on the changes in nuclear morphology (e.g., chromatin condensation and fragmentation).

### 4.6 Confocal raman microscopy of testicular sections

Raman analysis was performed using backscattering geometry in a confocal configuration at room temperature using a HR-800 Raman microscope system equipped with a 632.817 nm HeNe laser (JY Co., Fort-de-France, Martinique). It was reported that when the size of the TiO_2_ NPs reached 6 nm, the Raman spectral peak was 148.7 cm^−1^[74]. Laser power and resolution were approximately 20 mW and 0.3 cm^−1^, respectively, while the integration time was adjusted to 1 s. The testicular specimens (*n* = 5 in each group) were embedded in paraffin blocks, sliced into 5-μm thick sections, and placed onto glass slides. The slides were dewaxed, hydrated, and then scanned using the confocal Raman microscope.

### 4.7 Oxidative stress assay

Reactive oxygen species (ROS) (O_2_^**·−**^ and H_2_O_2_) production and levels of malondialdehyde (MDA), protein carbonyl (PC), and 8-hydroxy deoxyguanosine (8-OHdG) in the testicular tissues (*n* = 5 in each group) were assayed using commercial enzyme-linked immunosorbent assay kits (Nanjing Jiancheng Bioengineering Institute, Jiangsu, China) according to the manufacturer’s instructions.

### 4.8 Antioxidant capacity

The activities of superoxide dismutase (SOD), catalase (CAT), glutathione peroxidase (GPx), glutathione S epoxide transferase (GST), and glutathione reductase (GR), and the contents of reduced glutathione (GSH) and ascorbic acid in the testicular tissues (*n* = 5 in each group) were determined using commercial assay kits (Nanjing Jiancheng Bioengineering Institute, Jiangsu, China) according to the manufacturer’s instructions.

The article "Mechanisms of nanosized titanium dioxide-induced testicular oxidative stress and apoptosis in male mice" was retracted in 2015. Reasons: errors in the analysis; errors in the methods; duplicated images.

### 4.9 Assay of gene and protein expression

Total RNA was extracted from individual testes using from the homogenates was isolated using Tripure Isolation Reagent (Roche, USA) according to the manufacturer’s instructions. Probes and cycling condition were optimized in accordance with MIQE guidelines for PCR [75]. Synthesized cDNA was used for the real-time PCR by employing primers designed using Primer Express Software according to the software guidelines. PCR primers used in the gene expression analysis are listed in Table 3. Gene expression levels were calculated as a ratio to the expression of the reference gene, GAPDH and data were analyzed using the ΔΔCt method. The probes for SOD, CAT, GPx, GST, GR, Cyp1b1, carbonic anhydrase III (Car3), caspase-3, Bcl-2, nuclear receptor binding protein 2 (Nrbp2), acetyl-coenzyme A acyltransferase 2 (Acaa2), Axin upregulated 1 (Axud1), and cytochrome c were designed by the manufacturer and purchased from Shinegene Company (Shanghai, China). The RT-qPCR data were processed with the sequence detection software version 1.3.1 following the method of Schefe et al. [76].

**Table 3:** Real time PCR primer pairs

**Gene name**	**Description**	**Primer sequence**	**Primer size (bp)**
Refer- GAPDH	mactin-F	5′- TGTGTCCGTCGTGGATCTGA −3′	
	mactin-R	5′- TTGCTGTTGAAGTCGCAGGAG −3′	150
*SOD*	mSOD F	5′-CTGGACAAACCTGAGCCCTAA-3′	
	mSOD R	5′-TCCCCAGCAGCGGAATAA-3′	242
*CAT*	mCATF	5′-AGCGACCAGATGAAGCAGTG-3′	
	mCAT R	5′-GGGTGACCTCAAAGTATCCAAA-3′	241
*GSH-Px*	mGSH-Px F	5′-GGGACTACACCGAGATGAACG-3′	
	mGSH-Px R	5′-TCCGCAGGAAGGTAAAGAGC-3′	231
*GST*	mGST F	5′-CCGCTCTTTGGGGCTTTAT-3′	
	mGST R	5′-GGTTCTGGGACAGCAGGGT-3′	191
*GR*	mGR F	5′- TTCTGTTCATGGCGTGAGTACC −3′	
	mGR R	5′- CCCTTGGCACCTATTCCAGTT −3′	150
*Cyp1b1*	mCyp1b1-F	5′-TTAGTATGCTTTTCGCTGTGACA -3′	
	mCyp1b1-R	5′-GGGGAGTTATTCCTGGGTTATTA-3′	81
*Car3*	mcar3 F	5′-GCTCTGCTAAGACCATCC-3′	
	mcar3 R	5′-ATTGGCGAAGTCGGTAGG-3′	160 bp
*Caspase-3*	mcaspase-3 F	5′-CTGACTGGAAAGCCGAAACTC-3′	
	mcaspase-3 R	5′-GACTGGATGAACCACGACCC-3′	203
*Bcl-2*	mbcl-2 F	5′-TGTGGTCCATCTGACCCTCC-3′	
	mbcl-2 R	5′-ACATCTCCCTGTTGACGCTCT-3′	224
*Nrbp2*	mnrbp2 F	5′-TGCAGTGCAACCTGGAAA-3′	
	mnrbp2 R	5′-AGGAAACCAGGGTGGCTC-3′	188
*Acaa2*	macaa2 F	5′-TGTGTCAGAAATGTGCGCTTC-3′	
	macaa2 R	5′-CAAGGCGTATCTGTCACAGTC-3′	123
*Axud1*	mAxud1-F	5′-CGCCCTTCATTAGCTGATGTT -3′	
	mAxud1-R	5′-CAGAGCCTGCGTTTCTTGG-3′	117
*Cytochrome c*	mcytochrome c F	5′-CATCCCTTGACATCGTGCTT-3′	
	mcytochrome c R	5′-GGGTAGTCTGAGTAGCGTCGTG-3′	250

PCR primers used in the gene expression analysis.

To determine protein levels of SOD, CAT, GPx, GST, GR, Cyp1b1, Car3, caspase-3, Bcl-2, Nrbp2, Acaa2, Axud1, and cytochrome c in the testes, total protein from the frozen testicular tissues (*N* = 5 in each group) from experimental and control mice was extracted using Cell Lysis Kits (GENMED SCIENTIFICS INC.USA) and quantified using BCA protein assay kits (GENMED SCIENTIFICS INC.USA). ELISA was performed using commercial kits that were selective for each respective protein (R&D Systems, USA), following the manufacturer’s instructions. The absorbance was measured on a microplate reader at 450 nm (Varioskan Flash, Thermo Electron, Finland), and the concentrations of SOD, CAT, GPx, GST, GR, Cyp1b1, Car3, caspase-3, Bcl-2, Nrbp2, Acaa2, Axud1, and cytochrome c were calculated from a standard curve for each sample.

The article "Mechanisms of nanosized titanium dioxide-induced testicular oxidative stress and apoptosis in male mice" was retracted in 2015. Reasons: errors in the analysis; errors in the methods; duplicated images.

### 4.10 Statistical analysis

All results are expressed as means ± SD. One-way analysis of variance (ANOVA) was carried out to compare the differences of means among the multi-group data using SPSS 19 software (SPSS, Inc., Chicago, IL, USA). Dunnett’s test was performed when each dataset was compared with the solvent control data. Statistical significance for all tests was judged probability level of 0.05 (P < 0.05).

## Competing interests

The authors declare that they have no competing interests.

## Authors’ contributions

Conceived and designed the experiments: FH, XZ, LS, and LW. Performed the experiments: FH, XZ, LS, LW, JH, and XY. Analyzed the data: FH, XZ, LS, LW, JH, XY, YZ, XS, and QS. Contributed reagents/materials/analysis tools: YZ, XS, and QS. Wrote the paper: FH, XZ, LS, and LW. All authors read and approved the final manuscript.

## References

[B1] PowellJJFariaNThomas McKayEPeleLCOrigin and fate of dietary nanoparticles and microparticles in the gastrointestinal tractJ Autoimmun20103422623310.1016/j.jaut.2009.11.00620096538

[B2] WeirAWesterhoffPFabriciusLHristovskiKvon GoetzNTitanium dioxide nanoparticles in food and personal care productsEnviron Sci Technol2012462242225010.1021/es204168d22260395PMC3288463

[B3] FayazAMBalajiKGirilalMKalaichelvanPTVenkatesanRMycobased synthesis of silver nanoparticles and their incorporation into sodium alginate films for vegetable and fruit preservationJ Agric Food Chem2009576246625210.1021/jf900337h19552418

[B4] Lopez-Moreno ML, De La Rosa G, Hernandez-Viezcas JA, Peralta-Videa JR, Gardea-Torresdey JL: **X-ray absorption spectroscopy (XAS) corroboration of the uptake and storage of CeO**_**2**_**nanoparticles and assessment of their differential toxicity in four hdible plant species.***J Agric Food Chem* 2010, **58:**3689–3693.10.1021/jf904472ePMC285246020187606

[B5] GoutaillerGGuillardCFaureRPaïsséODegradation pathway of dicyclanil in water in the presence of titanium dioxide. Comparison with photolysisJ Agric Food Chem2002505115512010.1021/jf020294312188616

The article "Mechanisms of nanosized titanium dioxide-induced testicular oxidative stress and apoptosis in male mice" was retracted in 2015. Reasons: errors in the analysis; errors in the methods; duplicated images.

[B6] GimenoORivasFJBeltránFJCarbajoMPhotocatalytic ozonation of winery wastewatersJ Agric Food Chem2007559944995010.1021/jf072167i17960885

[B7] OberdörsterGOberdörsterEOberdörsterJNanotoxicology: an emerging discipline evolving from studies of ultrafine particlesEnviron Health Perspect2005113782383910.1289/ehp.733916002369PMC1257642

[B8] Wang JJ, Sanderson BJS, Wang H: **Cyto- and genotoxicity of ultrafine TiO**_**2**_**particles in cultured human lymphoblastoid cells.***Mutat Res* 2007, **628:**99–106.10.1016/j.mrgentox.2006.12.00317223607

[B9] Wang HH, Wick RL, Xing BS: **Toxicity of nanoparticulate and bulk ZnO, Al**_**2**_**O**_**3**_**and TiO**_**2**_**to the nematode caenorhabditis elegans.***Environ Pollut* 2009, **157:**1171–1177.10.1016/j.envpol.2008.11.00419081167

[B10] Xiong D, Fang T, Yu L, Sima X, Zhu W: **Effects of nano-scale TiO**_**2**_**, ZnO and their bulk counterparts on zebrafish: acute toxicity, oxidative stress and oxidative damage.***Sci Total Environ* 2011, **409**(8):1444–1452.10.1016/j.scitotenv.2011.01.01521296382

[B11] ShiHBMagayeRCastranovaVZhaoJSTitanium dioxide nanoparticles: a review of current toxicological dataPart Fibre Toxicol2013101510.1186/1743-8977-10-1523587290PMC3637140

[B12] OberdörsterGStoneVDonaldsonKToxicology of nanoparticles: a historical perspectiveNanotoxicol2007122510.1080/17435390701314761

[B13] LaZYangWXNanoparticles and spermatogenesis: how do nanoparticles affect spermatogenesis and penetrate the blood–testis barrierNanomed20127457959610.2217/nnm.12.2022471721

[B14] Komatsu T, Tabata M, Kubo-Irie M, Shimizu T, Suzuki KI, Nihei Y, Takeda K: **The effects of nanoparticles on mouse testis Leydig cells*****in vitro*****.***Toxicol in Vitro* 2008, **22:**1825–1831.10.1016/j.tiv.2008.08.00918805477

[B15] Hou J, Wan XY, Wang F, Xu GF, Liu Z, Zhang TB: **Effects of titanium dioxide nanoparticles on development and maturation of rat preantral follicle*****in vitro*****.***Acad J Second Military Med Univ* 2009, **30**(8):869–873 (In Chinese).

[B16] SuzukiHToyookaTIbukiYSimple and easy method to evaluate uptake potential of nanoparticles in mammalian cells using a flow cytometric light scatter analysisEnviron Sci Technol20074183018302410.1021/es062563217533873

[B17] Di VirgilioALReigosaMArnalPMFernández Lorenzo de MeleMComparative study of the cytotoxic and genotoxic effects of titanium oxide and aluminium oxide nanoparticles in Chinese hamster ovary (CHO-K1) cellsJ Hazard Mater201017771171810.1016/j.jhazmat.2009.12.08920079968

The article "Mechanisms of nanosized titanium dioxide-induced testicular oxidative stress and apoptosis in male mice" was retracted in 2015. Reasons: errors in the analysis; errors in the methods; duplicated images.

[B18] EmaMKobayashiNNayaMHanaiSNakanishiJReproductive and developmental toxicity studies of manufactured nanomaterialsReprod Toxicol201030334335210.1016/j.reprotox.2010.06.00220600821

[B19] TakedaKSuzukiKIshiharaAKubo-IrieMFujimotoRTabataMOshioSNiheiYIharaTSugamataMNanoparticles transferred from pregnant mice to their offspring can damage the genital and cranial nerve systemsJ Health20095595102

[B20] GuoLLLiuXHQinDXGaoLZhangHMLiuJYCuiYGEffects of nanosized titanium dioxide on the reproductive system of male miceZhonghua Nan Ke Xue200915517522(in Chinese)19593991

[B21] GaoGDZeYGLiBZhaoXYLiuXRShengLHuRPGuiSXSangXZSunQQChengJChengZWangLTangMHongFSThe ovarian dysfunction and its gene-expressed characteristics of female mice caused by long-term exposure to titanium dioxide nanoparticlesJ Hazard Mater2012243192710.1016/j.jhazmat.2012.08.04923131501

[B22] GaoGDZeYGZhaoXYSangXZZhengLZeXGuiSXShengLSunQQHongJYuXHWangLHongFSZhangXGTitanium dioxide nanoparticle-induced testicular damage, spermatogenesis suppression, and gene expression alterations in male miceJ Hazard Mater201325813314310.1016/j.jhazmat.2013.04.04623721730

[B23] SikkaSCRelative impact of oxidative stress on male reproductive functionCurr Med Chem2001885186210.2174/092986701337303911375755

[B24] MurugesanPMuthusamyTBalasbramanianKArunakarnJStudies on the protective role of vit-amin C and E against polychlorinated biphenyl (Aroclor 1254)-induced oxidative damage in Leydig cellsFree Radic Res2005391259127210.1080/1071576050030815416298753

[B25] GriveauJFDumontERenardPCallegariJPLannouDLReactive oxygen species, lipid-peroxdation and enzymatic defense systems in human spermatozoaJ Reprod Fert1995103172610.1530/jrf.0.10300177707295

[B26] HuJHZanLSZhaoXLLiQWJiangZLLiYKLiXEffects of tehalose supplementation on semen quality and oxidative varioables in frozen-thawed bovine semenJ Anim Sci2010881657166210.2527/jas.2009-233520081087

[B27] BaiYHZhangYZhangJPMuQXZhangWDButchERSnyderSEYanBRepeated administrations of carbon nanotubes in male mice cause reversible testis damage without affecting fertilityNat Nanotechnol2010568368910.1038/nnano.2010.15320693989PMC2934866

[B28] PryorWAHoukKNFooteCSFukutoJMIgnarroLJSquadritoGLDaviesKJAFree radical biology and medicine: it’s a gas, man!Am J Physiol Regul Integr Comp Physiol2006291R491R51110.1152/ajpregu.00614.200516627692

[B29] GuoLLLiuXHQinDXGaoLZhangHMLiuJYCuiYGStudy on the effect of nanosized zinc oxide for reproductive system of male miceJ Med Postgra201023357364(in Chinese)

[B30] YoshidaSHiyoshiKIchinoseTTakanoHOshioSSugawaraITakedaKShibamotoTEffect of nanoparticles on the male reproductive system of miceInt J Androl20083233734210.1111/j.1365-2605.2007.00865.x18217983

The article "Mechanisms of nanosized titanium dioxide-induced testicular oxidative stress and apoptosis in male mice" was retracted in 2015. Reasons: errors in the analysis; errors in the methods; duplicated images.

[B31] MorishitaYYoshiokaYSatohHNojiriNNaganoKAbeYKamadaHTsunodaSNabeshiHYoshikawaTTsutsumiYDistribution and histologic effects of intravenously administered amorphous nanosilica particles in the testes of miceBiochem Biophys Res Commun201242029730110.1016/j.bbrc.2012.02.15322417826

[B32] IavicoliILesoVFontanaLBergamaschiAToxicological effects of titanium dioxide nanoparticles: a review of in vitro studiesEur Rev Med Pharmacol Sci201115548150821744743

[B33] Iavicoli I, Leso V, Bergamaschi A: **Toxicological effects of titanium dioxide nanoparticles: a review of in vivo studies.***J Nanomater* 2012, 1–36. doi:10.1155/2012/964381.21744743

[B34] ZiniASchlegelPNCu/Zn superoxide dismutase, catalase and glutathione peroxidase mRNA expression in the rat testis after surgical cryptorchidism and efferent duct ligationJ Urol199715865966310.1016/S0022-5347(01)64578-69224387

[B35] IschiTMatsukiSIuchiYOkadaFToyosakiSTomitaYIkedaYFujiiJAccelerated impairment of spermatogenic cells in SOD1-knockout mice under heat stressFree Radic Res20053969570510.1080/1071576050013051716036348

[B36] MaiorinoMBoselloVUrsiniFForestaCGarollaAScapinMSztajerHFloheLGenetic varia-tions of GSH-Px-4 and male infertility in hum ansBiol Reprod2003681134114110.1095/biolreprod.102.00750012606444

[B37] CrawfordNMKahnMLLeustekTLongSRBuchanan BB, Gruissem W, Jones RLNitrogen and sulfurBiochemistry and molecular biology of plants2000ASPP, Rockville786849

[B38] SivoriJLCascorbic acidbeNZerbaENWoodEJInduction of glutathione S-transferase activity in Tria-tomainfestansMem Inst Oswaldo Cruz19979279780210.1590/S0074-027619970006000139566212

[B39] NarraVRHowellRWSastryKSRRaoDVVitamin C as a radioprotector against iodine-131 in vivoJ Nucl Med1993346376408455081

[B40] KutlubayROguzEOCanBGuvenMCSinikZTuncayOLVieamenEProtection from testicular damage caused by intraperitoneal aluminiumInt J Toxicol20072629730610.1080/1091581070147095217661220

[B41] ArmstrongJSSteinauerKKHornungBIrishJMLecanePBirrellGWPeehlDMKnoxSJRole of glutathione depletion and reactive oxygen species generation in apoptotic signaling in a human B lymphoma cell lineCell Death Differ2002925226310.1038/sj.cdd.440095911859408

[B42] SmirnoffNAntioxidants and reactive oxygen species in plants2005Blackwell Publishing, Oxford

[B43] Jovanović-GalovićABlagojevićDPGrubor-LajsićGWorlandRSpasićMBRole of antioxidant defense during different stages of preadult life cycle in European corn borer (Ostrinia nubilalis, Hubn.): Diapause and metamorphosisArch Insect Biochem Physiol2004552798910.1002/arch.1012614745825

[B44] AnguloCMaldonadoRPulgarEMancillaHCórdovaAVillarroelFCastroMAConchaIIVitamin C and oxidative stress in the seminiferous epitheliumBiol Res20114416918010.4067/S0716-9760201100020000922513420

The article "Mechanisms of nanosized titanium dioxide-induced testicular oxidative stress and apoptosis in male mice" was retracted in 2015. Reasons: errors in the analysis; errors in the methods; duplicated images.

[B45] KodamaHYamaguchiRFukudaJKascorbic acidiHTanakaTIncreased oxidative deoxyribonucleic acid damage in the spermatozoa of infertile male patientsFertl Steril19976851952410.1016/S0015-0282(97)00236-79314926

[B46] CuiYLGongXLDuanYMLiNHuRPLiuHTHongMMZhouMWangLWangHHongFSHepatocyte apoptosis and its molecular mechanisms in mice caused by titanium dioxide nanoparticlesJ Hazard Mater201018387488010.1016/j.jhazmat.2010.07.10920724067

[B47] GuiSXSangXZZhengLZeYGZhaoXYShengLSunQQChengZChengJHuRPWangLHongFSTangMIntragastric exposure to titanium dioxide nanoparticles induced nephrotoxicity in mice, assessed by physiological and gene expression modificationsPart Fibre Toxicol201310410.1186/1743-8977-10-423406204PMC3605279

[B48] Gui SX, Li BY, Zhao XY, Sheng L, Hong J, Yu XH, Sang XZ, Sun QQ, Ze YG, Wang L, Hong FS: **Renal injury and Nrf2 modulation in mouse kidney following chronic exposure to TiO**_**2**_**nanoparticles.***Agriic Food Chem* 2013, **61:**8959–8968.10.1021/jf402387e23968166

[B49] SunQQTanDLZhouQPLiuXRChengZLiuGZhuMSangXZGuiSXChengJHuRPTangMHongFSOxidative damage of lung and its protective mechanism in mice caused by long-term exposure to titanium dioxide nanoparticlesJ Biomed Mater Res Part A2012100A2554256210.1002/jbm.a.3419022528760

[B50] LiBZeYGSunQQZhangTSangXZCuiYLWangXCGuiSXTanDLZhuMZhaoXYShengLWangLHongFSTangMMolecular mechanisms of nanosized titanium dioxide–Induced pulmonary injury in micePlos One20138e5556310.1371/journal.pone.005556323409001PMC3567101

[B51] HuRPZhengLZhangTCuiYLGaoGDChengZChenJTangMHongFSMolecular mechanism of hippocampal apoptosis of mice following exposure to titanium dioxide nanoparticlesJ Hazard Mater2011191324010.1016/j.jhazmat.2011.04.02721570177

[B52] ChengCYMrukDDCell junction dynamics in the testis: Sertoli-germ cell interactions and male contraceptive developmentPhysiol Rev2002828258741227094510.1152/physrev.00009.2002

[B53] AlnemriESLivingstonDJNicholsonDWSalvesenGThornberryNAWongWWYuanJHuman ICE/CED-3 protease nomenclatureCell199687217110.1016/S0092-8674(00)81334-38861900

[B54] SalvesenGSCaspases: opening the boxes and interpreting the arrowsCell Death Differ2002913510.1038/sj.cdd.440096311803369

[B55] GhavamiSHashemiMAndeSRYeganehBXiaoWEshraghiMBusCJKadkhodaKWiechecEHalaykoAJLosMApoptosis and cancer: mutations within caspase genesJ Med Genet200946849751010.1136/jmg.2009.06694419505876

[B56] WaltersJPopCScottFLDragMSwartzPMattosCSalvesenGSClarkACA constitutively active and uninhibitable caspase-3 zymogen efficiently induces apoptosisBiochem J2009424333534510.1042/BJ2009082519788411PMC2805924

[B57] LiNDuanYMHongMMZhengLFeiMZhaoXYWangYCuiYLLiuHTCaiJWGongSJWangHHongFSSpleen injury and apoptotic pathway in mice caused bytitanium dioxide nanoparticulesToxicol Lett201019516116810.1016/j.toxlet.2010.03.111620381595

The article "Mechanisms of nanosized titanium dioxide-induced testicular oxidative stress and apoptosis in male mice" was retracted in 2015. Reasons: errors in the analysis; errors in the methods; duplicated images.

[B58] YangJLiuXSBhallaKKimCNIbradoAMCaiJPengTIJonesDPWangXPrevention of apoptosis by Bcl-2: release of cytochrome c from mitochondria blockedScience19972751129113210.1126/science.275.5303.11299027314

[B59] HowardSBottinoCBrookeSChengEGiffardRGSapolskyRNeuroprotective effects of Bcl-2 overexpression in hippocampal cultures: inter-actions with pathways of oxidative damageJ Neurochem20028391492310.1046/j.1471-4159.2002.01198.x12421364

[B60] StarkovAPolsterBFiskumGRegulation of hydrogen peroxide production by brain mitochondria by calcium and BaxJ Neurochem20028322022810.1046/j.1471-4159.2002.01153.x12358746

[B61] LarssonJForsbergMBrännvallKZhangXQEnarssonMHedborgFForsberg-NilssonKNuclear receptor binding protein 2 is induced during neural progenitor differentiation and affects cell survivalMole Cell Neurosci2008391323910.1016/j.mcn.2008.05.01318619852

[B62] CaoWLiuNSTangSBaoLShenLYuanHYZhaoXLuHAcetyl- Coenzyme A acyltransferase 2 attenuates the apoptotic effects of BNIP3 in two human cell linesBiochim Biophys Acta2008178087388810.1016/j.bbagen.2008.02.00718371312

[B63] GingrasSPelletierSBoydKIhleJNCharacterization of a family of novel cysteine-serine-rich nuclear proteins (CSRNP)Plos One200728e80810.1371/journal.pone.000080817726538PMC1950078

[B64] HsiehYGuanYTuCBrattPJAngerhoferJRLepockMHickeyMJTainerJANickHSSilvermanDNProbing the active site of human manganese superoxide disumtase: the role of glutamine 143Biochem1998374731473910.1021/bi972395d9537988

[B65] PonsESipilaPBritanAVernetPPoutaneriMHuhtaniemiIDrevetJRHinton BT, Turner TTEpididymal expression of mouse GSH-PX proteins: analysis of the mechanisms of GSH-PX5 tissue and region-specific expression through in vitro and in vivo approachesThird International Conference on the Epididymis2003The Van Doren Company, Charlottesville, VA7493

[B66] LiangHVan RemmenHFrohlichVLechleiterJRichardsonARanQGSH-Px4 protects mitochondrial ATP generation against oxidative damageBiochem Biophys Res Commun2007356489389810.1016/j.bbrc.2007.03.04517395155

[B67] ImaiHNakagawaYBiological significance of phospholipid hydroperoxide glutathione peroxidase (PHGSH-Px, GSH-Px4) in mammalian cellsFree Radic Biol Med200334214516910.1016/S0891-5849(02)01197-812521597

[B68] KimGLeeTHWetzelPGeersCRobinsonMAMyersTGOwensJWWehrNBEckhausMWGrosGWynshaw-BorisALevineRLCarbonic anhydrase III is not required in the mouse for normal growth, development, and life spanMol Cell Biol2004249942994710.1128/MCB.24.22.9942-9947.200415509796PMC525481

The article "Mechanisms of nanosized titanium dioxide-induced testicular oxidative stress and apoptosis in male mice" was retracted in 2015. Reasons: errors in the analysis; errors in the methods; duplicated images.

[B69] RaisanenSLehenkariPTascorbic AcidnenMRahikilaPHarkonenPLVaananenHKCarbonic anhydrase III protects cells from hydrogen peroxide-induced apoptosisFASEB J1999135135221006461810.1096/fasebj.13.3.513

[B70] TangYXScheefEAWangSJSorensonCMMarcusCBJefcoateCRSheibaniNCYP1B1 expression promotes the proangiogenic phenotype of endothelium through decreased intracellular oxidative stress and thrombospondin-2 expressionBlood2009113375175410.1182/blood-2008-03-145219PMC262838019005183

[B71] Yang P, Lu C, Hua N, Du Y: **Titanium dioxide nanoparticles co-doped with Fe**^**3+**^**and Eu**^**3+**^**ions for photocatalysis.***Mater Lett* 2002, **57:**794–801.

[B72] SangXZLiBZeYGHongJZeXGuiSXSunQQLiuHTZhaoXYShengLLiuDYuXHWangLHongFSToxicological mechanisms of nanosized titanium dioxide-induced spleen injury in mice after repeated peroral applicationAgric Food Chem2013615590559910.1021/jf303598923621103

[B73] TarabishyABAldabaghBSunYImamuraYMukherjeePKLassJHGhannoumMAPearlmanEMyD88 regulation of Fusarium keratitis is dependent on TLR4 and IL-1R1 but not TLR2J Immunol200818159360010.4049/jimmunol.181.1.59318566426PMC3909484

[B74] Zhang WF, He YL, Zhang MS, Yin Z, Chen Q: **Raman scattering study on anatase TiO**_**2**_**nanocrystals.***Phys D: Appl Phys* 2000, **33:**912–991.

[B75] BustinSABenesVGarsonJAHellemansJHuggettJKubistaMMuellerRNolanTPfafflMWShipleyGLVandesompeleJWittwerCTThe MIQE guidelines: minimum information for publication of quantitative real-time PCR experimentsClin Chem200955461162210.1373/clinchem.2008.11279719246619

[B76] SchefeJHLehmannKEBuschmannIRUngerTFunke-KaiserHQuantitative real-time RT-PCR data analysis: current concepts and the novel “gene expression’s CT difference” formulaJ Mol Med20068490191010.1007/s00109-006-0097-616972087

